The article "Big Transfer Learning for Fine Art Classification" was published in 2022. Journal: Comput Intell Neurosci.

# Big Transfer Learning for Fine Art Classification

**DOI:** 10.1155/2022/1764606

**Published:** 2022-05-31

**Authors:** Wentao Zhao, Wei Jiang, Xinguo Qiu

**Affiliations:** ^1^School of Intelligent Transportation, Zhejiang Institute of Mechanical & Electrical Engineering, Hangzhou 310053, Zhejiang, China; ^2^College of Mechanical Engineering, Zhejiang University of Technology, Hangzhou 310023, Zhejiang, China

## Abstract

Automatic classification and retrieval of fine art collections have received much attention in recent years. In this article, we explore the applicability of convolutional neural networks (CNNs) for art-related image classification tasks. To examine how hyperparameters affect model performance, we use different hyperparameters in our experiments and find that a higher resolution and appropriate training steps with mix-up can improve model performance. To determine how transfer learning affects the final results, we systematically compare the efforts of five weight initializations of the models for different tasks. We show that fine-tuning networks pretrained on a larger dataset have better generalizability. This phenomenon shows the a priori knowledge that models learn in the real world also applies to the art world, and we call this method as big transfer learning (BiT). Through extensive experiments on fine art classification, we demonstrate that the proposed transfer learning approach outperforms the previous work by a large margin and achieves state-of-the-art performance in the art field. Furthermore, to show how computers capture features in paintings to make classifications, we visualized the results of different classification tasks to help us understand the operation mechanism of the models. Additionally, we use our models to retrieve paintings by analyzing different image similarity aspects. The results show that models can be employed to retrieve paintings even if they are computer-generated.

## 1. Introduction

The number of fine art collections that have been digitized has increased rapidly in recent years. To manage and index these vast collections, we must classify, index, and retrieve paintings. Art experts can identify the artist, genre, style, and some other metadata of paintings using their experience. However, this manual work is time-consuming and requires history and art experts. Therefore, the automatic recognition of artworks' characteristics can not only generate the existing metadata such as artist, genre, and style in new collections but also create new metadata types related to the artwork's content or specific stylistic characteristics [1, 2].

Consequently, many studies have been conducted to investigate how to teach a computer to understand various painting characteristics. Research progress in the domain of fine art classification has also made great progress recently by large and well-annotated fine datasets [3], and recent breakthroughs in computer vision achieved by deep convolutional neural networks (CNNs) [4, 5]. More datasets, from small to large, have been introduced in the art field for different tasks, Painting-91 [6], the Rijksmuseum Challenge Dataset [7, 8], WikiArt [9], ART500K [10, 11], the OmniArt dataset [12], and the newly introduced MultitaskPainting100k dataset [13]. In addition, datasets such as SemArt [14, 15] and BibleVSA [16] are introduced to perform visual-semantic retrieval [17]. The use of a large dataset makes it possible to use CNNs for fine art classification tasks [3, 18, 19].

One of the main recent successes of deep CNNs is the use of pretraining parameters trained with extra labeled out-of-domain data, such as ILSVRC-2012 [20], which contains 1.3 M images, ImageNet-21k [21], which contains 14 M images, and JFT [22], which contains 300 M images [23]. Compared with these large public datasets, digitized paintings are still limited, and it is difficult to train a generalized model without overfitting. Excellent performance has been achieved in many different image-related classification tasks in many fields by fine-tuning CNNs pretrained on the ImageNet dataset [24–26]. This research inspires us to explore how transfer learning works on fine-art-specific tasks such as artist, genre, and style recognition.

In our work, we explore how transfer learning affects fine art recognition performance. Our contributions are as follows:

- We use different training schedule lengths and resolutions without mix-up to test the impact on the final results and find that a higher resolution and appropriate training steps with mix-up can improve model accuracy.
- We use 5 weight initialization methods in the models, with both pretrained in-domain and out-of-domain data, to explore the impact of weight initialization. We show that the pretrained weight initialization method influences the fine-tuning performance. By using models pretrained on a larger dataset, the model has better generalizability. The model will perform better if it is fine-tuned in a larger art dataset first.
- We compare our results with those of previous work. This comparison shows that our results obtain state-of-the-art results in all tasks with different datasets. Furthermore, we evaluate the performance with little downstream data and find that it still works well in the specific task.
- We visualize and analyze some phenomena worth attention. The results show that one of the reasons for misclassification was the similar elements or painting styles among the paintings.
- We build a painting retrieval system based on the trained classification models. It shows that models can be used to retrieve content-based searches across art datasets with both existing paintings and computer-generated paintings.

## 2. Related Work

Automatic art classification is a basic research topic in painting computational aesthetics. Early work in automatic art analysis first extracted handcrafted features from the images and performed classification using traditional machine learning methods [27–29]. For example, Falomir et al. [30] presented QArt-Learn approach for style painting categorization using the k-nearest neighbor and support vector machine methods with quantum chromodynamics (QCD) color features and quantitative global features. Saleh and Elgammal [31] explored how different features and metric learning approaches influence the classification results and achieved the best results with the feature fusion method. Zhong et al. [32] used the RGB and brush stroke information to classify fine art painting images. In recent years, deep CNNs have achieved great success in computer vision using large hand-labeled datasets such as the ImageNet dataset [20]. The research is mainly carried out through a model structure selection, data augmentation, feature fusion, and transfer learning [33]. Model structure selection means optimizing the model structure to improve model performance in art classification. Zhao et al. [34] compare the performance of different models that have made great success in ImageNet recently for art classification. Sandoval et al. [19] introduced a two-stage image classification approach including a deep CNN and a shallow neural network to improve the style classification accuracy. For the data augmentation, Badea et al. [35] used the Sun database [36] to augment some WikiArt classes and used ResNet-34, which was not initialized on ImageNet, to perform genre classification tasks. Feature fusion means incorporating expert knowledge into automatic feature models. Chu and Wu [37] learned deep correlation features (LDCF) from Gram and obtained 64.32% and 78.27% in artist and style classification tasks, respectively, in Painting-91. Bianco et al. [13] proposed the MultitaskPainting100k dataset and used a spatial transformer network (STN), which was introduced by [38] with the injection of histogram of oriented gradient (HOG) features to achieve accuracies of 56.5%, 63.6%, and 57.2% in artist, genre, and style tasks, respectively. Chen and Yang [39] presented an end-to-end trainable architecture including adaptive cross-layer correlation, and the results show it can adaptively weight features in different spatial locations.

Transfer learning aims at transferring the trained model parameters to a new model training. A well-established paradigm has been to pretrain models using larger-scale data and then to fine-tune the models on the specific tasks [40–42]. Tan et al. [9] achieved the best results by fine-tuning AlexNet pretrained on the ImageNet dataset. Viswanathan [43] use ResNet-18 with pretrained weights from the ImageNet dataset in artist classification tasks. Cetinic et al. [44] used a fine-tuned CaffeNet pretrained on domain-specific datasets and achieved the best performance. The average accuracy for the artist, style, and genre classification tasks obtained through the most advanced methods is described in Section 3.3. From the aforementioned studies, for specific tasks in art classification, transfer learning is generally performed using the ILSVRC-2012 version of ImageNet [21] or domain-specific datasets for model pretraining. To fill this gap regarding pretraining only with ILSVRC-2012, we pretrained the model on a larger dataset, ImageNet-21K [23] to further enhance the pretraining performance. Furthermore, we evaluated the influence of hyperparameters and downstream dataset size on the effectiveness of transfer learning to obtain a better transfer learning method and improve the model performance for art classification.

In addition to attribute prediction, Ypsilantis et al. [45] built the Met dataset for Instance-Level Recognition (ILR) in the artwork domain. Zhao et al. [46] used artistic comments to classify painting attributes and find word embeddings can be used to explain the meaning of the label.

## 3. Materials and Methods

### 3.1. Datasets

With the aim of classifying paintings, we use three different datasets to identify the artist, genre, and style classification tasks. Our first source is Painting-91 [6], which is a small dataset used for analyzing digital paintings. This dataset contains 4,266 images from 91 different painters. In total, 2,338 paintings have been labeled with the style to which the painting belongs. The styles used in this study are as follows: Abstract Expressionism, Baroque, Constructivism, Cubism, Impressionism, Neoclassicism, Pop Art, Post-Impressionism, Realism, Renaissance, Romanticism, Surrealism, and Symbolism. This dataset is widely used because the categories of artist and style are distributed uniformly and is convenient for training due to its small size. Another large-scale dataset is WikiArt-WikiPaintings, which is collected from WikiArt [31]. The nonprofit painting art website and painting art are shared and annotated by volunteers. As the number of paintings on websites increases over time, the painting screening methods of different papers are different, so the number of paintings and the number of categories among algorithms are different. For a fair comparison, we use the dataset as Tan et al. [9] set. More than 80,000 fine art paintings are collected from WikiArt, including more than 1,000 artists, 27 different styles, and 45 different genres. Then, we use a limited number of samples available in some classes for the tasks. In the end, all the paintings are used for style classification; only 10 genres with more than 1,500 paintings are chosen for genre classification, and 23 artists with more than 500 paintings are used for artist classification. The distribution of per class in each task can be seen in Figure 1. Furthermore, we explore another source of paintings-MultitaskPainting100k. The dataset comes from the Painter by Numbers Kaggle competition, which predicts whether a pair of images are from the same artist or not. It contains 103,250 images of paintings mainly from WikiArt. The rest of the paintings are provided by the artists specifically for competition. Then, classes are removed with fewer than 10 entries in each task. After selection, 99,816 paintings for 1,508 artists, 125 styles, and 41 genres are used in the dataset. Different from WikiArt-WikiPaintings, each image record includes 3 attributes, allowing every image to be used for artist, style, and genre classification tasks. The distribution of categories is more uneven, which means that some categories have only a small number of images, which makes the classification tasks more difficult. In our experiments, we use the same data splitting scheme to fairly compare with previous studies. Larger training datasets contain more painting diversity and can enhance model generalization. The total number of images per task and dataset, including the training/testing split and the number of classes, is provided in Table 1. Examples of representative images from three different data sources are shown in Figure 2.

### 3.2. Model Selection

The models used in our experiment are ResNet-50 with ResNet-v2 architecture [47], which is modified from ResNet [48]. We use group normalization [49] instead of batch normalization [50] and add weight standardization [51] to all the convolutional layers. To research how transfer learning works in the art domain using external data, we use the initialized parameters pretrained on CIFAR-10 [52], ILSVRC-2012, ImageNet-21k [23], and the in-domain dataset MultitaskPainting100k.

### 3.3. Training Setting

The pseudocode of fine-tuning the CNN and obtaining the accuracy can be seen in Algorithm 1. In each iteration, we randomly sample *b* images to compute the gradients and then update the network parameters. Instead of limiting the training epochs, we limit the training steps. For hyperparameter selection, we use stochastic gradient descent (SGD) [53] with an initial learning rate of 0.03, a momentum of 0.9, and a batch size of 64. In general, a larger training set size can significantly improve the generalization of the model. Makantasis et al. [54–57] reduced the number of weight parameters by making the parameter weights satisfy rank-1 canonical decomposition, which in turn reduces the required training samples. Here, for the data augmentation, we first resize a larger image to 512 × 512, take a random crop to 480 × 480, then make random horizontal flips, and normalize them in the training data. We resize to 480 directly and normalize the test data. For the schedule length, we use 500 steps in Painting-91 and 10,000 steps in WikiArt and MultitaskPainting100k. During fine-tuning, we first warm up and then decay the learning rate 3 times by a factor of 10 at some steps of the training steps (see Section 4.2). Finally, we use mix-up (1) with *λ*=0.1 in all the tasks in the WikiArt and MultitaskPainting100k datasets to perform data augmentation, as shown in Algorithm 1:

(1) $$\begin{array}{c} \left\{\begin{array}{c} \tilde{x}=\lambda x_{i}+\left(1-\lambda \right)x_{j},\\ \tilde{y}=\lambda y_{i}+\left(1-\lambda \right)y_{j}, \end{array}\right) \end{array}$$

where *x*_*i*_ and *x*_*j*_ are the raw input vectors and *y*_*i*_ and *y*_*j*_ are the labels. Then, we obtain the new vectors and labels. The loss function is defined using the cross-entropy loss function:

(2) $$\begin{array}{c} \mathrm{loss}\left(x,\text{class}\right)=-\log\left(\frac{\exp\left(x\left[\text{class}\right]\right)}{\sum_{j}\exp\left(x\left[j\right]\right)}\right)\\ =-x\left[\text{class}\right]+\log\left(\sum_{j}\exp\left(x\left[j\right]\right)\right), \end{array}$$

where *x* ∈ *ℝ*^*N*×*C*^ is the output of the models, class ∈ *ℝ*^*N*^ is the label of the painting, and 0 ≤ class[*i*] ≤ *C* − 1.

## 4. Results and Discussion

In this section, we evaluate our fine-tuning strategy on 3 different tasks in 3 datasets. We want to answer the following questions:

- How do different hyperparameters, including the resolution, training schedule length, and whether to use mix-up regulation, affect the art classification results?
- How do different weight initializations trained from the out-of-domain and in-domain data affect the final result in each task?
- Can our model achieve satisfactory results in art classification, even with limited labeled data?
- How can a painting retrieval system be built, and how does it perform using painting embeddings to retrieve paintings?

### 4.1. Test Performance

We run our experiments using the training setting as shown in Section 3.3, and the results of each task are summarized in Tables 2–4, together with the results of previous state-of-the-art approaches measured on the datasets. BiT-S and BiT-M are pretrained on ILSVRC-2012 and ImageNet-21k, respectively. The WikiArt datasets are both from the WikiArt website, and as the number of paintings on websites increases over time, there are differences in the selection methods of paintings for different studies, so the number of paintings and number of categories are different among the algorithms. We also report the number of classes and samples considered in the experiments presented in each paper in Table 3. Although the dataset configurations are not exactly the same, because the data are from the same source, they still have a certain reference value. MultitaskPainting100k has 2 versions: the original version and resizing to 256. We use these 2 versions and find that the original images obtain higher performance (68.14%, 65.82%, 72.64%) (Table 4). This finding proves that a compressed image uses interpolation to enlarge the image loses much information. All related works have been described in Section 2 and compared to the references above, and all of our models achieve state-of-the-art performance. Note that we use fewer epochs and do not perform a hyperparameter grid search, which means that it still has room for improvement and proves how important it is for weight initialization pretrained on a large, generic dataset.

### 4.2. Parameter Sensitivity

We explore the test accuracies with different hyperparameters for the artist, style, and genre classification tasks: the training schedule length, resolution, and whether to use mix-up. For both the training schedule length and resolution, we use 4 kinds of combinations. For painting resolution, we set (160, 128), (256, 224), (448, 384), and (512, 480). The former represents the resized size in the training phase, while the latter represents the random cropping size in the training and testing phases. Due to the different input image resolutions, the floating point operations (FLOPs) of the model are 1.35 GFlops, 4.13 GFlops, 12.14 GFlops, 18.97 GFlops, respectively. For the training schedule length, we use [100, 200, 300, 400, 500], [500, 1,500, 3,000, 4,500, 5,000], [500, 3,000, 6,000, 9,000, 10,000], and [500, 6,000, 12,000, 18,000, 20,000]. The first parameter means the warm-up steps, the last is the end step, while the others mean steps in which the learning rate decays by a factor of 10.  Figure 3 shows the test accuracy for different resolutions and training schedule lengths without mix-up. We can see that using a higher resolution can increase the recognition accuracy, which means that clearer paintings carry more information. A longer training schedule length can also increase the accuracy, but when longer than 10,000, the effect is not obvious. This indicates that too long training schedule length can cause overfitting of the model training. Using mix-up can improve the performance in the artist and genre recognition task, but it has no effort in the style classification task, and models perform worst in style classification. This finding shows that the task of identifying painting styles is challenging for computers.

### 4.3. Impact of Weight Initialization

To evaluate how weight initialization affects task performance, we use the pretrained ResNet50 model to explore how upstream pretraining affects the fine-tuning performance:

- BiT-M is trained on the full ImageNet-21k dataset, a public dataset containing 14.2 M images and 21K classes organized by the WordNet hierarchy. Images may contain multiple labels.
- BiT-S is trained on the ILSVRC-2012 variant of ImageNet, and it contains 1.28 M images and 1,000 classes.
- BiT-M-S is trained on the ImageNet-21k dataset and then fine-tuned on ILSVRC-2012.
- BiT-M-C is trained on the ImageNet-21k dataset and then fine-tuned on CIFAR-10, which contains 60,000 32 × 32 color images in 10 classes, with 6,000 images per class.
- BiT-M-Mul is trained on the ImageNet-21k dataset and then fine-tuned on MultitaskPainting100k.

The first 4 weight initialization models are out-of-domain data and from Kolesnikov et al. [23]. The last are in-domain data and trained by us. To make a fair comparison, we set the schedule to 10,000 steps and use mix-up regulation. The other settings are the same as those in Section 3.3. The results for the weight initialization impact are shown in Table 5. We find that models pretrained on ImageNet-21k have a better generalization performance than those pretrained on ILSVRC-2012. Even fine-tuning in the out-of-domain datasets does not hurt the generalizability. Models fine-tuned on art datasets can improve their generalizability in painting classification tasks. We calculate the test performance every 100 stages and plot the graph as shown in Figure 4. It can be found that BiT-M-Mul performs best in different stages of training. This finding proves that weight initialization using in-domain data achieves an excellent performance. Because there are many identical images between MultitaskPainting100k and WikiArt, we do not use the result of BiT-M-Mul as the final result, but it still has reference significance. The models pretrained on ImageNet-21k (BiT-M, BiT-M-S, and BiT-M-C) perform better in most of the training steps compared with weight initialization using ILSVRC-2012 (BiT-S). This finding shows that larger datasets have better generalizability, although they are not as effective as pretraining in the field.

### 4.4. Effect of the Size of the Labeled Data

To evaluate the model performance in small downstream data, we randomly select the number of images per class and test the performance.  Figure 5 is an example of a randomly selected 5-shot WikiArt dataset. The low data performance is shown in Figure 6. The *X*-axis is the number of images per class. The blue bars show fine-tuning on the full dataset, the orange bars show the state-of-the-art results from previous work, and the green bars show fine-tuning on the models pretrained on ILSVRC2012. We note that BiT-M can achieve a higher test accuracy with limited labeled images in WikiArt. For instance, BiT-M achieves a test accuracy of 42.31% with only 5 images per genre. When each category contains 100 images, the models achieve accuracies of 84.77% and 68.74% in the artist and genre classification tasks, respectively. Due to the large number of categories and the small number of paintings in each category, the classification performance of models in MultitaskPainting100k is not outstanding. Our model achieves state-of-the-art performance in all the tasks in these 2 datasets. This finding proves that pretraining plays an important role in classification tasks.

### 4.5. Interpretation of the Classification Results

Figure 7 shows the embedding of paintings using fine-tuned BiT-M models. There are a few observations that are worth attention combined with Figure 8(c). Categories such as abstract paintings, landscapes, and portraits are clustered, which makes these categories well distinguished, similar to the excellent performance of CNNs in face detection and scene recognition. These paintings achieve 95%, 90%, and 86% recognition rates in each category, respectively. The paintings belonging to sketches and studies are confused with other types of paintings, which results in an accuracy of only 66% for these types of paintings. Upon further examination of Figure 8(c), cityscapes are mistaken for landscapes because they all include outdoor scenes; illustrations and nude paintings are often referred to as genre paintings because they all contain people, which can also be seen in Figure 5. Regarding style classification (Figure 8(b)), we can observe that the most obvious type of style is Ukiyo-e (96%), which is a genre of woodblock prints and paintings that flourished in Japan from the late 17th to late 19th centuries. Action Painting was a style widespread from the 1940s until the early 1960s and is closely associated with Abstract Expressionism. This style is difficult for computers to distinguish because of the relationship between the two contains and is contained, and nearly half of the Action Paintings are predicted as Abstract Expressionist paintings. Synthetic Cubism (58%) and Analytical Cubism (70%) are easy to categorize into Cubism because Analytical Cubism and Synthetic Cubism are the two key phases of Cubism. From the style analysis above, we can also see that inadequate datasets, Analytical Cubism, and Synthetic Cubism are the different stages of Cubism. Action and Color Field painting are 2 substyles of Abstract Expressionism based on 2 different ways of applying color. It can be seen that the model performs best in the artist classification task (Figure 8(a)). Pablo Picasso's (84%) artistic career runs through almost his entire life, and his work is often categorized into periods, which makes his works rich and diverse. However, it makes it difficult for the models to distinguish his artwork. Ivan Aivazovsky (99%) was a Russian Romantic painter and is considered one of the greatest masters of marine art. The vast majority of his works are seascapes. Raphael Kirchner (99%) was a famous postcard painter and is best known for Art Nouveau. The content of his paintings is often sweet and colorful girls and gorgeous life as the background. Rembrandt (99%) was a Dutch painter; Rembrandt lighting, which was named for him, is often used in his paintings. We can find that the artists that models can recognize with high precision usually use certain objects or technologies in their paintings. These findings are in line with the results of Tan et al. [9]. This finding shows that the recognition mechanism of the model for paintings is basically the same. However, after using a higher painting resolution and better model pretrained using a larger dataset and other methods, our classification accuracy is higher than that of this previous work.

### 4.6. Feature Extractor for Image Similarity

In addition to exploring task-specific classification, we aimed at retrieving the paintings of similar categories. To accomplish the retrieval goal, we used various models to perform feature extraction and then calculated the similarity between features using the cosine distance. We use paintings from different sources as the input and search for similar paintings in terms of artist, style, and genre from MultitaskPainting100K. For each of them, we retrieved the 6 most similar paintings using artist, style, and genre features. The Young Ladies of Avignon (Figure 9) is a large oil painting created in 1907 by the Spanish artist Pablo Picasso. It depicts five nude female prostitutes in a brothel, and the three figures on the left exhibit facial features in the Iberian style of Picasso's native Spain, while the two figures on the right are shown with African mask-like features. This incredible painting marked not only a major turning point in Picasso's personal art history but also a revolutionary breakthrough in the history of Western modern art, which marks the birth of Cubism. Only 4 of 6 paintings belonging to Pablo Picasso were retrieved by the system using artist features. It also shows difficulty recognizing the artists who have different painting styles because we know Picasso was a prolific painter and his works were rich and varied in style from Section 4.5. Because portraits and nude paintings (nu) all have human bodies, when retrieving genres, some portrait paintings were also retrieved. In total, it performed well in style and genre retrieval. Berendey's Sloboda (Figure 10) (which does not belong to the MultitaskPainting100k dataset) was painted by Nicholas Roerich, who was a Russian painter, writer, archaeologist, theosophist, philosopher, and public figure. We can obtain the correct retrieval use only the genre. It is difficult to distinguish the author and style very well even for adults who have less experience in art. It shows that sketches and studies are difficult to classify especially in terms of the artist and style due to the single color. This phenomenon also verifies why the recognition rate of sketches and studies is the lowest in genre classification. DeepArt is a website that allows users to create unique artist images in the style of your favorite artist by using transfer learning [60]. Here, we use Lenna, which is a standard test image widely used in the field of image processing since 1973, as the source image and van Gogh's self-portrait as the style source to create a new image and feed it to the retrieval system in Figure 11. Van Gogh is one of the greatest of the Post-Impressionists, and the eye-catching colors, prominent brushstrokes, and outline forms in his works have strongly influenced the trend of modern artistic expressionism. Interestingly, all 3 of the most similar paintings retrieved by the system using artist features are from Vincent van Gogh, and the first is just the painting as the style source. All 6 paintings retrieved using the style and genre features belong to the Post-Impressionism style and portrait genre, similar to the style source image. This shows that this system is still very useful for computer-generated images.

## 5. Conclusions

In this study, we use transfer learning and fine-tuning on 3 art collections for 3 different art-related classification tasks. We focus on exploring the impact of different weight initializations and show that the pretrained model influences the fine-tuning performance. Moreover, we show that pretraining on ImageNet21k yields a better generalizability. Our approach achieves a state-of-the-art performance in all the tasks in the 3 datasets compared with previous work. In addition, we build an image retrieval system that provides similar paintings with respect to artist, style, and genre features, which helps users better understand the paintings. The retrieval results show that this system works well not only on existing paintings but also on computer-generated paintings. In this work, we used convolutional neural networks (CNNs) to perform various types of artwork classifications. In a given set of paintings, the artists, styles, genres, and other features may be related to each other. For example, van Gogh's paintings have a high probability of being classified as Post-Impressionist, as he was the greatest Post-Impressionist. Therefore, in future work, we will attempt to add other features to construct classification approaches based on both color features and contextual relationships between labels. In Section 4.5, we found problems with dataset tags, such as Action Paintings for Abstract Expressionism and Analytical Cubism and Synthetic Cubism for Cubism. Therefore, it is necessary to build a more comprehensive and in-depth painting dataset and consider both quantity and quality. Also, we will further explore the effect of different convolutional kernels and convolutional network sizes in art classification.

## Figures and Tables

**Figure 1:** Class distribution of the WikiArt in each task. (a) WikiArt artist distribution. (b) WikiArt genre distribution. (c) WikiArt style distribution.

**Figure 2:** Examples of images from the three data sources. (a) Painting91. (b) WikiArt. (c) MultitaskPainting100k.

**Figure 3:** Test accuracy with different hyperparameters.

**Figure 4:** Validation accuracy curves of differently initialized models for the WikiArt artist, style, and genre classification tasks: (a) Artists. (b) Styles. (c) Genres.

**Figure 5:** The whole 5-shot WikiArt dataset in the genre classification task.

**Figure 6:** Test accuracy by varying the number of images per class in the training data. (a) WikiArt. (b) MultitaskPainting100k.

**Figure 7:** Embedding of the paintings projected in WikiArt using t-SNE [58]. Each node is a painting, and the coloring is mapped to the genre attribute. The meaning of the colors can be seen in the figure legend.

**Figure 8:** Confusion matrix [59] for WikiArt artist, style, and genre classification tasks using the Bit-M fine-tuned model. The color bar shows the normalized intensity. (a) Artists. (b) Styles. (c) Genres.

**Figure 9:** Similarity results for the young ladies of Avignon by Pablo Picasso, belonging to the cubism style and nude painting (nu) genre. Similarity results: the top 6 paintings retrieved using the artist features (first row), style features (second row), and genre features (third row).

**Figure 10:** Similarity results for Berendey's Sloboda by Nicholas Roerich. Similarity results: the top 6 paintings retrieved using the artist features (first row), style features (second row), and genre features (third row).

**Figure 11:** Similarity results for Lenna using van Gogh's self-portrait, which belongs to the Post-Impressionist style, and the portrait genre as the style source. Similarity results: the top 6 paintings retrieved using the artist features (first row), style features (second row), and genre features (third row).

**Algorithm 1:** Fine-tuning the neural network and obtaining the painting classification accuracy.

**Table 1:** Number of images and classes for the different sources and tasks.

Source	Task	Class	Train	Test	Total
Painting-91	Artist	91	2,275	1,991	4,266
	Style	13	1,250	1,088	2,338

WikiArt	Artist	23	13,344	5,706	19,050
	Genre	10	45,501	19,492	64,993
	Style	27	57,023	24,421	81,444

MultitaskPainting100k	Artist	1,508	69,821	29,995	99,816
	Genre	41	69,821	29,995	99,816
	Style	125	69,821	29,995	99,816

**Table 2:** State-of-the-art results for artist and style categorization on the Painting-91 dataset.

Reference	Method	Painting-91		
		Artist	Style	Average
[37]	LDCF (learned from gram)	64.32	78.27	71.30
[39]	Cross-layer correlation	70.65	78.13	74.39
[34]	Structure selection	71.27	79.23	75.25
BiT-S (ours)	Big transfer learning	61.23	75.64	68.44
BiT-M (ours)	Big transfer learning	**72.07**	**79.60**	**75.84**

The bold values show that the proposed BiT-M model achieves state-of-the-art performance compared with previous work and BiT-S model.

**Table 3:** State-of-the-art results for artist, genre, and style categorization on the WikiArt dataset, including samples and classes in each task.

Reference	Year	Method	Artist			Style			Genre		
			Sample	Classes	Acc. (%)	Samples	Classes	Acc. (%)	Samples	Classes	Acc. (%)
[9]	2016	CNN fine-tuning (AlexNet)	19,050	23	76.11	81,444	27	54.5	64,993	10	74.14
[31]	2016	Feature fusion	18,599	23	63.06	78,449	27	45.97	63,691	10	60.28
[43]	2017	CNN fine-tuning (ResNet18)	17,100	57	77.7						
[35]	2017	CNN fine-tuning (ResNet-34)							79,434	26	61.15
[44]	2018	CNN fine-tuning (CaffeNet)	20,320	23	81.94	96,014	27	56.43	86,087	10	77.6
[19]	2019	Two-stage classification approach				26,400	22	66.71			
[32]	2020	RGB and brush stroke channels	9766	19	88.38	30,825	25	58.99	28,760	10	76.27
[34]	2021	Structure selection	19,050	23	91.73	81,444	27	69.97	64,993	10	78.03
BiT-S (ours)		Big transfer	19,050	23	91.34	81,444	27	68.27	64,993	10	80.88
BiT-M (ours)		Big transfer	19,050	23	**93.50**	81,444	27	**71.24**	64,993	10	**82.39**

The bold values show that the proposed transfer learning approach outperforms the previous work by a large margin and achieves state-of-the-art performance in the art field.

**Table 4:** State-of-the-art results for artist, genre, and style categorization on the original MultitaskPainting100k dataset and the resized one.

Reference	Method	MultitaskPainting100k			
		Artist	Style	Genre	Average
[13]	STN + HOG	56.5	57.2	63.6	56.85
[34]	Structure selection	65.50	63.15	67.83	65.49
BiT-S (ours)	Big transfer-256	51.38	60.16	70.23	55.77
BiT-M (ours)	Big transfer-256	66.04	64.32	71.97	65.18
BiT-S (ours)	Big transfer-ori	53.72	61.12	70.48	61.77
BiT-M (ours)	Big transfer-ori	**68.14**	**65.82**	**72.64**	**68.87**

**Table 5:** Comparison of the classification accuracies achieved with different initializations.

Weight initialization	Tasks/acc. (%)			Average
	Artist	Style	Genre	
BiT-M	94.01	71.49	82.07	82.52
BiT-S	91.45	67.88	80.57	79.97
BiT-M-C	93.88	71.59	82.13	82.53
BiT-M-S	93.94	71.31	81.80	82.35
BiT-M-Mul	**95.20**	**75.78**	**84.52**	**85.17**

It shows BiT-M-Mul model achieves state-of-the-art performance compared with other weight initialization models.

## Data Availability

Painting-91 is available at https://www.cat.uab.cat/∼joost/painting91.html. WikiArt is available at https://github.com/cs-chan/ArtGAN. MultitaskPainting100K is available at https://www.ivl.disco.unimib.it/activities/paintings.
